# Influence of Three-Dimensional Visual Reconstruction Technology Combined with Virtual Surgical Planning of CTA Images on Precise Resection of Liver Cancer in Hepatobiliary Surgery

**DOI:** 10.1155/2022/4376654

**Published:** 2022-07-07

**Authors:** Yuanyu Zhao, Ting Chen, Hui Wang, Qiang Xue, Wenyuan Guo, Guoshan Ding, Junfeng Dong, Junsong Ji

**Affiliations:** ^1^Department of Liver Surgery, Changzheng Hospital, Naval Medical University, Shanghai 200003, China; ^2^Department of General Surgery, Shanghai Jing'an District Zhabei Central Hospital, Shanghai 200070, China; ^3^Department of Neurosurgery, Eastern Hepatobiliary Surgery Hospital, Navy Medical University, Shanghai 200082, China

## Abstract

Hepatobiliary malignancies, such as hepatocellular carcinoma (HCC) and biliary tract cancers, namely, gallbladder carcinoma and cholangiocarcinoma, are linked to a high rate of morbidity and mortality, depending on the phase of the disease. The intricate hepatobiliary anatomy and the need for accurate peroperative management, especially in patients with advanced liver disease, make these tumors difficult to treat. Surgical resection is a notable therapy for hepatobiliary cancers. Unnecessary or excessive liver excision influences patient rehabilitation, normal liver function, and postoperative complications. Hepatobiliary operations must therefore include accurate liver removal. The present advancements in imaging technology are aimed at improving the diagnostic efficacy of liver injury even more. Three-dimensional visual reconstruction is becoming more important in the diagnosis as well as treatment of a variety of disorders. In this paper, we proposed a novel three-dimensional visual reconstruction technology using enhanced nonuniform rational basis spline (ENURBS) combined with virtual surgical planning of Computed Tomography Angiography (CTA) images for precise liver cancer resection. The purpose of this project is to rebuild 2D CTA scan images of liver cancer into a 3D reconstructed model for efficient visualization and diagnosis of liver cancer and to prepare an effective preoperative surgical plan for precise liver excision based on a 3D recreated liver model. This method's performance is compared to that of 2D planning in terms of accuracy and time taken to complete the plan. It is concluded that our proposed technique outperforms the planning technique based on 2D images.

## 1. Introduction

One of the most dangerous diseases is liver cancer, often known as hepatic cancer. Hepatitis B and C viruses, fatty liver illness, drug-related cirrhosis, glowing, fatness, diabetes, iron overburden, and different dietary hazards are all prominent causes of HC. Liver cancer is the most common reason for cancerous deaths worldwide and the 5^th^ most prevalent in the US, and it is one of the top 5 dangerous malignancies to experience a yearly proportion increase in occurrences [1]. HCC has been the most prevalent kind of liver cancer, responsible for roughly 80% of all occurrences [2]. Nearly 78 percent of the 600,000 instances of HCC are noted worldwide in Asian countries. Chronic hepatitis B virus disease is the major source of HCC in Eastern Asia.

In the complete medication of liver disease, surgical resection (removal of the cancerous segment in the organ) remains supreme. It has the potential to cure patients with better efficiency and to extend the overall survival duration of those who undergo surgery. Liver resection is a significant, life-threatening procedure that should only be performed by surgeons with extensive experience. The major concern for surgeons is the selection of the correct tumor segment for liver resection from the 2D medical images such as CT, MRI, CTA, and X-ray because of the complexities in the analysis of hepatobiliary anatomy. Computed Tomography Angiography (CTA) is an imaging technique that combines injection of contrast material into the blood vessel with a CT scanner to produce cross-sectional pictures of soft tissue, skeletal anatomy, and vascular frames. 3D images reduce the complexities in the analysis of hepatic anatomy.

Doctors previously used their personal knowledge to transform 2D scan images into an abstract 3D model. Nonetheless, the reconstruction conclusion may be incorrect and inconsistent due to the limitations and ambiguities of their experience [7]. As a result, utilizing computer-aided software or mathematical models to digitally reconstruct 3D images from 2D photographs could be a viable solution to the aforementioned dilemma. Three-dimensional visual reconstruction (3DVR) is becoming more and more important in the analysis and cure of liver illnesses [8]. Although 3D rebuilt or 3D printing technology designs may visually represent intrahepatic blood vessel changes, they also include an efficient and comfortable approach for liver volume estimation, virtual simulation operation, and operative guidance [9]. 3D viewing includes extraction of features and 3D reconstruction of CT/MRI/CTA images utilizing modern computing techniques. It is a method of seeing, describing, and evaluating 3D anatomy and morphological properties of organs in order to make more intuitive, realistic, and reliable medical decisions [10].

When surgical treatments are preceded by proper planning, the results are usually better. Proper planning of liver resection which includes the examination of precise tumor segment that must be excised is required because unnecessary liver resection has an impact on patient recovery, surgical complications, and liver function [11]. To provide optimal treatment, it is critical to visualize the lesion to be treated directly or indirectly from the 3D reconstructed image. Virtual surgical planning (VSP) is quickly becoming a standard of care for even the most complex surgeries [12].

In this research, we proposed a new enhanced three-dimensional visual reconstruction technology-enhanced nonuniform rational basis spline (ENURBS) combined with virtual surgical planning of CTA images on precise resection of liver cancer in hepatobiliary surgery. The first focus of this work is to reconstruct the 2D CTA images of liver cancer into 3D reconstructed model using the ENURBS algorithm for efficient visualization and diagnosis of liver cancer. The second goal is to plan the surgical methods using VSP based on the 3D reconstructed liver model for precise liver resection. The performance of this approach is compared with that of 2D images.

The further organizations of the research paper are shown below.  Section 2 shows the problem statement.  Section 3 provides the flow of the proposed work. Performance evaluation is given in Section 4. Finally, Section 5 gives the conclusion of the proposed paper.

## 2. Problem Statement

Liver disease is a major risk to human life, so it was among the most internal cancers in the world, as well as one of the principal factors of cancer-related death. Hence, efficient diagnosis and proper treatment are the major concerns in curing the patients. Diagnosis using 2D CTA images of the liver is very complicated and time-consuming for surgeons because of the complex hepatic structure. So there is a need for modern imaging techniques. One such technique is a 3D visual reconstruction from 2D images which provides a clear visualization of liver anatomy and improves the surgeon's knowledge. Surgical resection is the prominent treatment for preventing the further dispersal of liver tumors and curing the patients. Choosing an optimal approach for liver resection is a critical task before treatment because unnecessary liver resection has an impact on patient recovery and normal liver function. Hence, advanced preoperative surgical planning before surgical intervention is required for removing precise liver tumor segments and improving the efficiency of treatment. By considering these factors, we proposed three-dimensional visual reconstruction technology combined with virtual surgical planning of CTA images on precise resection of liver cancer in hepatobiliary surgery.

## 3. Proposed Work

In this section, we define the dataset, image processing, 3D reconstruction-virtual surgical planning, ENURBS algorithm, 3D reconstruction of the hepatic centerline, 3D reconstruction of the hepatic cross section, 3D reconstruction of the hepatic surface, and planning of surgical methods in detail.

Accurate liver resection is very significant for a better outcome in curing patients with liver cancer. Three-dimensional visual reconstruction technology combined with virtual surgical planning is used in this work. The 2D CTA images of liver cancer are preprocessed at first. Then, the images are reconstructed into a 3D image using ENURBS for efficient visualization and diagnosis of liver cancer. Finally, planning of the surgical methods based on the 3D reconstructed liver model for precise liver resection is performed using VSP. The flow of the proposed work is shown in Figure 1 and explained in this section.

### 3.1. Dataset

In our study, we used the clinical dataset that was prescribed in [6]. The dataset consists of six CTA volumes of the abdomen imaged at the portal venous region, among which two volumes are pathologic. Every dataset volume is made up of a sequence of 2D CT layers with a quality of 512∗512 axial planes as well as a width of 0.5–2 mm. Every volume has a different quantity, ranging between 212 and 395.

### 3.2. Image Preprocessing

Noise removal and node and segment labeling are included in the image preprocessing of 2D CTA liver images. The presence of noise in an image can reduce image quality, further complicating the image processing process [13]. As a result, to increase image quality, undesirable noises must be removed. A hybrid median filter was employed to remove noises such as impulsive and Gaussian disturbances. With the use of the Gaussian distribution, Gaussian smoothing is accomplished in conjunction with a median filter. The median filter uses the Gaussian distribution and medians to remove noisy pixels or noise without affecting edges or minute details. Each component of the image is recreated using the preprocessed photo elements [14]. The final stage is to improve image quality to obtain a high-quality image for future diagnostics and processing [15].

The Gaussian distribution *R*_(*b*)_(*A*) is determined by

(1) $$\begin{array}{c} R_{\left(b\right)}\left(A\right)=\frac{1}{\sigma {\sqrt{2\pi }}^{e}}e^{-{\left(A-\mu \right)}^{2}/2\sigma^{2}}, \end{array}$$

where *μ* is the mean and *σ* denotes the standard deviation.

The median of the image pixels is *y*[*m*, *n*] by

(2) $$\begin{array}{c} y\left[m,n\right]={\text{median}}_{\left(u,v\right)\in k_{xy}\left\{g\left(u,v\right)\right\}}, \end{array}$$

where *k*_*xy*_ are the coordinate sets centered at the point (*x*, *y*).

2D liver borders are eliminated employing a fast marching level set technique on the CTA abdominal picture by characterizing liver borders as the reproducing front final location. The vascular centerline is determined using a subvoxel precise skeletonization method. The centerline can be computed as the cheapest path between an ending point and a beginning point by performing a gradient descent over the fast marching distance map.

Given a 2D image of the skeleton of a liver structure, nodes (that is, branching points) and segments were discovered and labeled on each projection using the binary image's connection matrix. An eight-connectivity seed-fill technique was used to find connected pixels. The seed-fill technique began with a center point and explored its neighbors iteratively to find related facts [16]. Labels may propagate differently depending on the projection. The insertion points for liver removal are used to verify label correspondence. These points were marked to ensure that they were consistent among forecasts. The Euclidean distance was used to match an insertion point to a node. Only nodes with the same initialization point were kept. As a result, node labels and branching across projections were guaranteed to match.

### 3.3. 3D Reconstruction-Virtual Surgical Planning

The proposed technique involves reconstruction of the 3D image from the 2D CTA image using the ENURBS 3D approach and planning of the surgical methods based on the 3D reconstructed liver model for precise liver resection using VSP.

### 3.4. ENURBS Algorithm

The major steps involved in our proposed algorithm are as follows:

- 3D reconstruction of the hepatic centerline
- 3D reconstruction of the hepatic cross section
- 3D reconstruction of the hepatic surface

Using this algorithm, a 3D reconstructed CTA liver image will be generated from the preprocessed 2D CTA image.

### 3.5. 3D Reconstruction of the Hepatic Centerline

A 3D vascular centerline was created by intersecting surfaces defined by comparable liver segments. The segment correspondences between two projection planes *P*_*n*_ and *P*_*m*_ were estimated. Let the pair of transformed liver centerlines be *X*_*n*_ and *X*_*m*_ and their corresponding focal points be *F*_*n*_ and *F*_*m*_. The surfaces *R*_*n*_ and *R*_*m*_ representing the projection beams for *X*_*n*_ and *X*_*m*_ were produced by connecting the centerlines and focal points. The issue of identifying the 3D centerline (*C*) in the curves *X*_*n*_ and *X*_*m*_ can be mitigated to the identification of the intersection line of the 2 surfaces *R*_*n*_ and *R*_*m*_, as given in

(3) $$\begin{array}{c} C=R_{m}\cap R_{n}. \end{array}$$

*R*_*n*_ and *R*_*m*_ were triangulated surfaces, and the fast mutual triangle intersection testing was used to calculate their intersection. If two triangles meet, they lap over at the intersection line of their various planes, according to this analysis. In a nutshell, the test determines the signed range between a triangle's three vertices in the plane comprising another triangle. The two triangles do not intersect if all of the distances have the same sign. Otherwise, they may meet, reducing the problem to a two-segment overlap test on the junction line. The algorithm determines whether scalar gaps within each triangle have an intersecting path; if they do, the intersecting line segment that would be the two separate places is determined [17]. Construction difficulties can develop whenever the triangles are mostly coplanar or even when one border is approximately coplanar to another triangle. To handle such scenarios, a tolerance valuation for the ranges between vertices of two triangles has been determined by noticing the greatest 3D Euclidean distance with both relating sights attained experimentally; that is, if a tip is fairly similar to the plane of other triangles, it is taken into account to be on the plane. The crossings between 2 triangulated fields produced an organized number of attributes, which were linked to form a 3D midline.

### 3.6. 3D Reconstruction of the Hepatic Cross Section

The 3D cross sections were produced by keeping the 3D generated centerline as the base. The collection of accessible projection lines, their mutual alignment, and their direction concerning the liver section of interest affect the precision of the liver contour in 3D reconstruction from CTA. In CTA images, there are few *N* projection planes. Based on these findings, a 3D cross section was built in two stages: initially, an estimate was employed to deal with a limited set of projections, and then, the original cross section was localized in line with 2D liver borders.

At equidistant places “*a*” along a 3D rebuilt centerline curve, cross-sectional planes were formed in 3D space. With a 3D point (*x*_*a*_, *y*_*a*_, *z*_*a*_) on *C*, a cross-sectional plane *R*_*a*_ was determined with the help of tangential vector $\hat{m_{R_{a}}}$of *C* at (*x*_*a*_, *y*_*a*_, *z*_*a*_). The 2D image point (*u*_*a*,*m*_, *v*_*a*,*m*_) is the point of projection (*x*_*a*_, *y*_*a*_, *z*_*a*_) on the projection plane *P*_*m*_. The diameter vector which is orthogonal to the direction of the 2D liver centerline at (*u*_*a*,*m*_, *v*_*a*,*m*_) was *D*_*a*,*m*_. The magnification factor (M.F), which was derived using equation (4), was then applied to expand this vector.

(4) $$\begin{array}{c} \text{M}.\text{F}=\frac{\left(x_{a},y_{a},z_{a}\right)}{D\left(F_{m},\right.\left(u_{a,m},v_{a,m}\right)}. \end{array}$$

The diameter vector was not always orthogonal to *C* at (*x*_*a*_, *y*_*a*_, *z*_*a*_). Hence, the expanded diameter *D*_*a*,*m*_^*N*^ is imposed on the plane of the cross-sectional plane at (*x*_*a*_, *y*_*a*_, *z*_*a*_). A liver contour was developed as a circle at this point, with a diameter equal to the average length of rebuilt diameter vectors *D*′_*a*,*m*_ given in

(5) $$\begin{array}{c} D\prime_{a,m}=D_{a,m}^{N}-\left(D_{a,m}^{N}.\hat{m_{R_{a}}}\right)\hat{m_{R_{a}}}. \end{array}$$

To parametrize a liver contour, the nonuniform rational basis spline (NURBS) mechanism was applied. The creation of a flexible and versatile cross-section modeling utilizing NURBS parameterization, which can express simple curves like circles as well as more complex free-form curves, is performed. The determination of liver contour is given in

(6) $$\begin{array}{c} \gamma_{a}\left(u\right)=\overset{m}{\underset{i=0}{\sum }}B_{i,p}\left(u\right)Q_{i}u\in \left[0,1\right], \end{array}$$

where *n* + 1 represents the total number of used control points, “*Q*_*i*_” denotes the control points, *p* is the curve's degree, and *B*_*i*,*p*_(*u*) is a function defined on the knot vector of the *i*^th^ control points and *p*^th^ degree, which is dependent on a rational basis.

The circular contour *γ*_*a*_(*u*) was first sampled evenly along its path, and the curve's order was three. The control points were uniformly dispersed along their length. The curve's shape was then tweaked as follows. A pair of 3D axial points used for the description of the 3D liver cross section at (*x*_*a*_, *y*_*a*_, *z*_*a*_) is generated for each plane by equation (5). Let *N* represent the overall planes of projection. Then, *Q*_*a*_ = 2 N points which denote the 3D liver cross sections of the liver were produced.

For the liver contour *γ*_*a*_(*u*), 3D points *Q*_*a*_ were tagged as interpolatory control points. The Euclidean distances were calculated from the control points *γ*_*a*_(*u*) for each *Q*_*a*_. Every point *Q*_*a*_ replaced its nearest point. The multiplicity of a point's knot value was enhanced to attain interpolation. A knot value was inserted continuously till its multiplicity attains the curve's degree. Noninterpolatory control points were designated on the remaining control points.

### 3.7. 3D Reconstruction of the Hepatic Surface

To construct the 3D surface of a liver scan traversing through a collection of liver contours, a technique known as lofting or skinning can be used. The new control points *s* of the lofted vessel surface were obtained by interpolating over the control points in each liver contour. Some attention was made to maintain liver surface continuity before interpolation over contours. To ensure that the liver surface did not flip or twist, control points were sorted according to their angles on the plane and in the same direction (clockwise). Furthermore, every starting control point of contours established a continuous curve; without this precaution, torsion regions in the liver surface would appear according to the curve discontinuities [18].

The curves also had to be suitable, which means that they should have the identical number of control points and degrees; also, they should be described on the identical knot vector. Knot vectors were merged, degrees were raised to their peak value, and knots were placed by which all contours will have identical knot vector and control points. These steps are conducted for ensuring compatibility. This procedure did not affect the structure of the liver outlines.

The knot vector “*V*” was estimated, and it is applied to interpolate degree-*q* curves *γ*_*i*_(*v*) through the control points by

(7) $$\begin{array}{c} \gamma_{i}\left(v\right)=\overset{n}{\underset{j=0}{\sum }}B_{j,p}\left(v\right)P_{j}. \end{array}$$

As a result, equation (8) interpolated *Q*_*i*_ at different *v* values.

(8) $$\begin{array}{c} G\left(u,v\right)=\overset{m}{\underset{i}{\sum }}\overset{n}{\underset{j}{\sum }}B_{i,p}\left(u\right)B_{j,q}\left(v\right)P_{i,j}. \end{array}$$

These newly discovered control points are the lofted surface that is the hepatic surface and control points specified across the knot vectors *U* and *V*. As shown in equation (8), 3D liver surfaces were recreated using the lofting technique.

By integrating the results of the above three steps, a 3D reconstructed liver image was obtained. The liver cross-sectional areas of the resultant 3D reconstructed segment were computed using Stokes theorem for determining the area of a planar polygon. On a liver cross-sectional curve, parametric points *p*_*i*_ given by equation (9) were generated using a uniform distribution.

(9) $$\begin{array}{c} \left\{p_{i}=\left(u_{i},v_{i}\right)\right\},\;\text{i}=0,\cdots .,n. \end{array}$$

The area *A* contained by the curve was calculated by

(10) $$\begin{array}{c} A=\frac{1}{2}\overset{m}{\underset{i=0}{\sum }}\left(u_{i}V_{\left(i+1\right)}-u_{\left(i+1\right)}V_{i}\right.. \end{array}$$

### 3.8. Planning of Surgical Methods

Virtual surgical planning is used to plan liver resections, which includes detecting precise tumor portions that must be removed for effective treatment (VSP). VSP is a preoperative planning approach that involves visualizing a surgical procedure in a computer or virtual environment and developing a realistic plan using 3D reconstructed models. The steps in VSP are as follows.

Once the 3D reconstructed liver image is obtained, a VSP meeting with a biomedical engineer or a 3D designer and the surgical team is held online. 3D models are further expanded to produce cutting guides and the custom plate based on surgical needs for resection (e.g., clear margins from tumors and viable tissue in osteonecrosis) and reconstruction (e.g., number of segments following osteotomies). Before surgery, the stereolithographic recipient and donor models, liver cutting guides, fixation guide, and virtual reconstructed liver model are 3D printed, tested, and changed as needed. The final models are 3D printed and sterilised before the surgery. If a custom-made titanium plate is possible, it is built and sent along with the printed model; if not, a reconstruction plate is installed.

The following parameters are considered in 3D visualization in VSP:

- Examination of lesions in the hepatic region of the 3D model based on the attributes such as shape, size, and location of lesions and the study of the structural connection between lesions and intrahepatic arteries
- Morphological analysis of the arterial system in the hepatic area
- Detection of the venous system of the liver
- Structural examination of the portal venous segment of the liver
- Liver segmentation and calculation of liver volume. To segment and compute the liver volume, the structural relationship of blood flow in portal veins is used. In the meantime, the volume of drainage area in any branch of the portal vein branch is determined. Volume predictions are also required for significant liver resections and living liver donations. Initially, the 3D classification method shown in Table 1 is according to [4]. This aids surgeons in assessing the liver parts for resection in VSP. The optimal plane of virtual resection is estimated depending on the location of the tumor and the spatial relationship and distance between the intrahepatic vascular system and the region of the tumor. The volume of the functional liver that remains is determined using simulation surgery. In the meantime, the postoperative integrity of drainage and blood supply of hepatic veins in each hepatic segment retained should be ensured

## 4. Results and Discussion

3D reconstruction of the 2D CTA liver image taken from the dataset was performed using the ENURBS algorithm, and then, preoperative planning of the surgical method was done using VSP. This section deals with the simulation results and their detailed explanation. The influence of our approach on liver resection was evaluated based on the performance metrics such as accuracy and prediction time. Simulation graphs were obtained using MATLAB.  Figure 2 shows the sample of a 3D reconstructed liver tumor model of a 2D CTA image considered from the dataset.

From Figure 3, it is shown that the accuracy of visualizing the precise tumor segment from the 3D reconstructed liver model using ENURBS is higher than that of 2D CTA images. Figure 1 shows that surgeons can more precisely visualize the tumor section from the 3D reconstructed model than from 2D images. Our findings suggest that 3D reconstruction increases clinicians' ability to create the best surgical strategy.

Comparative analysis of the performance of the surgical planning methods based on 2D images and our proposed method is shown in Table 2.  Figure 4 shows the accuracy of the surgical plans generated by the above-mentioned two approaches. The proposed ENURBS-VSP method generates the surgical plan for liver resection with higher accuracy compared to that generated based on 2D scan reports.  Figure 5 depicts that the time taken to complete the overall surgical plan using the proposed VSP technique was significantly lesser compared to that taken by the 2D planning method. Hence, it is concluded from the simulation results that 3DVR using the ENURBS approach integrated with VSP can provide a proper and accurate preoperative plan before surgical liver intervention in a short period. Using this plan, the excision of a precise tumor segment from the whole liver organ can be achieved. So patients with liver cancer can effectively be treated.

## 5. Conclusions

Liver cancer is one of the most significant fatal malignancies all over the world. Surgical intervention is the prominent treatment for curing liver cancer. The advancements in digital intelligent screening and treatment technologies have promoted the efficiency of liver surgery. In this paper, we combined 3D visual reconstruction of CTA liver images using the ENURBS 3DVR technique with virtual surgical planning in liver cancer resection. The goal of this research is to use precise removal of liver tumor segments to cure patients more quickly and reduce operation time. According to the simulation results, 3DVR with ENURBS paired with VSP can provide a proper and accurate preoperative plan before surgical liver intervention in a short amount of time. With this plan, a specific tumor part can be excised from the complete liver organ. Hence, people with liver cancer can be treated efficiently. In the future, this study must be extended to a larger dataset. In addition, extensive postoperative investigations on the patient's health and liver functionality must be conducted.

## Figures and Tables

**Figure 1:** Detailed flow of the proposed work.

**Figure 2:** 3D reconstructed liver model.

**Figure 3:** Accuracy of the 3D reconstructed model.

**Figure 4:** Accuracy of surgical planning techniques.

**Figure 5:** Average time taken to finish the plan by different techniques.

**Table 1:** 3D visualization classification of HCC.

Classification description	Surgical methods
Type I: lesions are identified in the parenchyma of liver segments V and VIII or both segments and are distinguished by their closeness to, or even direct violation of, the next portal vein. They do not cling to the right hepatic vein trunk or compress it	Excision of liver segments V and VIII ± partial intervention of segment IV

Type II: lesions are located in the parenchyma of hepatic segments IVa and IVb or both segments and are distinguished by their proximity to, or even direct violation of, the left hepatic vein branch. Furthermore, it does not attach to or compress the trunk of the left hepatic vein	Excision of liver segments IVa and IVb or left hepatectomy

Type III: most of the liver parenchyma in segments IV, V, and VIII is occupied by the lesions, which is characterized by a wide and deep invasion of the parenchyma, as well as proximity to the main hepatic vein	Central bisectionectomy (removal of segments IV, V, and VIII±I)

Type IV: most liver parenchyma in segments IV, V, and VIII is occupied by lesions, which is distinguished by its closeness to, or direct violation of, the left/right portal vein branch or the left/right hepatic vein.	Excision of segment IV, V, VI, VII, and VIII removal reduced right trisectionectomy or reduced left trisectionectomy Associating liver partition and portal vein ligation for staged hepatectomy (ALPPS)

Type V: the superficial liver parenchyma of segments IV, V, and VIII is occupied by this form of liver tumor. Neither the portal branch nor the hepatic vein is near the lesions	Hepatectomy with a negative margin

**Table 2:** Comparative analysis of the performance of 3D and 2D approaches.

Approaches	Average time for completing the plan (s)	Accuracy of the plan (%)
Surgical planning based on 2D images	86	65
ENURBS-VSP technique (proposed)	70	85

## Data Availability

The analyzed datasets generated during the study are available from the corresponding author upon request.
